RETRACTED

# MRI Diagnosis and Pathological Examination of Axillary Lymph Node Metastasis in Breast Cancer Patients

**DOI:** 10.1155/2022/4519982

**Published:** 2022-09-14

**Authors:** Xiaodan Fu, Bingjing Jiang, Jieting Fu, Jinli Jia

**Affiliations:** ^1^Pathology Department, Affiliated Jinhua Hospital, Zhejiang University School of Medicine, Jinhua 321000, China; ^2^Imaging Department, Affiliated Jinhua Hospital, Zhejiang University School of Medicine, Jinhua 321000, China

## Abstract

In order to explore the characteristics and diagnostic value of magnetic resonance imaging (MRI) in axillary lymph node metastasis of breast cancer, a total of 200 breast cancer patients diagnosed and treated from January 2021 to January 2022 are selected as the study subjects, and 200 patients are divided into an axillary lymph node metastasis group and a simple breast cancer group according to pathological results. The pathological results are used as the gold standard to determine the accuracy and diagnostic efficacy of MRI results. A multivariate logistic regression method is used to analyze the influencing factors of MRI image characteristics of breast cancer axillary lymph node metastasis. The experimental results show that MRI has high application values in diagnosing axillary lymph node metastasis of breast cancer, which is worthy of clinical promotion and application.

## 1. Introduction

Breast cancer is a malignant tumor disease with a high incidence in women, which is characterized by high mortality, atypical symptoms, and easy metastasis, posing a serious threat to women's life and health [1]. The primary focus and lymph node metastasis have a serious impact on the therapeutic effect and prognosis of breast cancer patients. Surgical resection and lymph node cleaning are the main treatment of axillary lymph nodes, preoperative accurately predicting axillary lymph node properties of disease staging, treatment, and curative effect evaluation [2]. Lymph node biopsy pathological examination is the gold standard for checking the properties of axillary lymph nodes, but it is an invasive examination and can cause complications such as pain, lymphedema, and dyskinesia. Imaging examination is a commonly used auxiliary technology for clinical disease diagnosis and lesion examination. Magnetic resonance imaging (MRI) is the nucleus after image reconstruction processing in the magnetic resonance signal of imaging technology, but the value of application in the axillary lymph node metastasis of breast cancer is still unknown [3, 4]. The purpose of this study is to calculate and analyze the characteristics and diagnostic value of MRI imaging parameters in axillary lymph node metastasis of breast cancer with pathological examination as the gold standard so as to provide a new direction for the imaging diagnosis of axillary lymph node metastasis of breast cancer in the later stage.

RETRACTED

The rest of this paper is organized as follows: Section 2 discusses related work.  Section 3 discusses magnetic resonance imaging and data analysis. The pathological examination and univariate analysis are discussed in Section 4.  Section 5 concludes the paper with summary.

## 2. Related Work

Breast cancer [5] is the malignant disease threat to women's health, and axillary lymph node cleaning could obtain a certain effect but would increase in patients with upper limb nerve damage and the risk of complications such as lymphedema, so the prognosis assessment had an important influence [6]. MRI technology had the advantage of high tissue resolution, and the combination of the gradient echo imaging sequence and the paramagnetic contrast agent could obtain accurate results in the pathological staging diagnosis of breast cancer [7, 8].

Dave et al. [9] pointed out that the location of breast cancer would affect axillary lymph node metastasis. The maximum diameter of lymph nodes in patients without metastasis was significantly smaller than that in patients with axillary lymph node metastasis and was a risk factor for axillary lymph node metastasis, suggesting that patients with large diameter lymph nodes had a higher risk of metastasis. Gong et al. [10] indicated that the smaller the diameter of the lymph node, the lower the risk of lymph node metastasis, which might be due to the increased pulmonary vascular infiltration and lymph node tissue in patients with larger diameter tumors.

Both the distribution of intravascular contrast agents and the early enhancement mode could sensitively reflect the microvascular density and specific distribution of the body [11]. It was speculated that the main mechanism was as follows: breast cancer primary tumors of hemodynamic changes would affect axillary lymph node metastasis. Blood supply was rich, the higher the degree of structure specificity of a malignant tumor, the greater the risk of shift, and there was a higher risk of axillary lymph node metastasis [12].

## 3. Magnetic Resonance Imaging and Data Analysis

A total of 200 breast cancer patients admitted to our hospital from January 2021 to January 2022 are selected as the study subjects. All patients underwent surgical treatment and preventive lymph node dissection. According to the final pathological results, all patients are divided into an axillary lymph node metastasis group and a simple breast cancer group. The average age is (41.79 ± 2.32) years. There are 38 males and 162 females, 67 cases of drinking history and 90 cases of smoking history. The included subjects are diagnosed with breast cancer by cytology, imaging, and postoperative pathological examination, and their clinical data and surgical records are complete. At the same time, ipsilateral lymph node dissection is performed, and the expected survival time is more than 3 months. Patients whose location and type of lymph node metastasis could not be determined according to pathological results are excluded; patients who have received radiotherapy and chemotherapy such as sunitinib, docetaxel, and cisplatin before participating in the study or who have taken other anticancer drugs within the recent 30 days are excluded; patients with other malignant tumors and abnormal mental state are excluded.

RETRACTED

A GE Signa HDxt 3.0 T magnetic resonance instrument and an 8-channel phased front coil are used for MRI examination. MRI was performed in prone position and the breast was placed in the coil hole. MRI plain scan parameters are set as follows: layer thickness is 4.0 mm, layer spacing is 5 mm, TR and TE parameters are 8200 ms and 36.72 ms. Repetition time (TR) and echo time (TE) parameters are 400 ms and 7.82 ms. The parameters of diffusion-weighted imaging (DWI) are 0, B is set to 1000 s/m m2, and TR and TE are set to 6378 ms and 69.8 ms, respectively. Gd-dtpa is injected with a high pressure syringe at a rate of 0.1 mmol/kg through the median cubital vein. The tube is rinsed with 10 ml of normal saline, and the dynamic-enhanced scan is performed. The parameters of AXI GR are 4.33 ms and 2.10 ms, and a total of 8 stages were performed.

The obtained image data are transmitted to an ADW 4.3 workstation, and the apparent diffusion coefficient (ADC) of mammary axillary lymph nodes is measured by function tool software. The data are measured by two or more attending physicians and averaged. The criteria for axillary lymph node metastasis are as follows: axillary lymph node metastasis is confirmed by medical examination before and after surgery.

SPSS 22.0 software is used to complete effective processing of the data presented in the study. The measurement data are tested for normality and homogeneity of variance to satisfy normal distribution. The mean ± standard deviation ($\bar{x}$ ± *s*) is used to represent the data, and the *t*-test is performed. A multivariate logistic regression method is used to analyze the influencing factors of the MRI image. According to the characteristics of axillary lymph node metastasis of breast cancer, the specificity and sensitivity of MRI in diagnosing axillary lymph node metastasis of breast cancer were obtained.

## 4. Pathological Examination and Univariate Analysis

Table 1 shows the results of pathological examination and MRI examination. It is clearly evident from Table 1 that MRI detects 102 cases of axillary lymph node metastasis, 98 cases without axillary lymph node metastasis, 10 cases of false positive, and 8 cases of false negative. The accuracy is 91.00%.

RETRACTED

Table 2 shows the diagnostic efficacy of MRI in breast cancer with axillary lymph node metastasis. It is clearly evident from Table 2 that AUC is greater than 0.9, and sensitivity and specificity are greater than or equal 90.00%.

Figure 1 shows the diagnostic ROC curve of axillary lymph node metastasis in breast cancer by MRI. It is clearly evident from Table 1 that ROC is greater than 0.8.

Table 3 shows the univariate analysis of the associations between breast cancer MRI findings and axillary lymph node metastasis. It is clearly evident from Table 3 that there are significant statistical differences in MRI locations between the axillary lymph node metastasis group and the simple breast cancer group, and the proportion of the outer quadrant of the axillary lymph node metastasis group is higher (*P* < 0.05). There is no significant difference in the type of breast cancer between the axillary lymph node metastasis group and the simple breast cancer group (*P* > 0.05).

Table 4 shows the univariate analysis of the relationship between MRI features of breast lump-like lesions and axillary lymph node metastasis. It is clearly evident from Table 4 that in the group with axillary lymph node metastasis, MRI edge irregularity, proportion of early rapid enhancement, and maximum mass diameter are higher than those in the group with simple breast cancer, and ADC values are lower, with statistically significant differences (*P* < 0.05). There are no significant differences in MRI morphology and internal enhancement between the axillary lymph node metastasis group and the simple breast cancer group (*P* > 0.05).

Table 5 shows the variable assignment table. It is clearly evident from Table 5 that *P* is less than 0.05.

Table 6 shows the multivariate logistic regression analysis of MRI imaging characteristics in breast cancer with axillary lymph node metastasis. It is clearly evident from Table 6 that the risk factors for breast cancer axillary lymph node metastasis include the maximum diameter, outer quadrant, irregular edge, and early rapid enhancement.

Figure 2 shows the multivariate logistic regression analysis of the characteristics of axillary lymph node metastasis in breast cancer. It is clearly evident from Figure 2 that the ADC value is a protective factor, and the early reinforcement mode is 2.651.

RETRACTED

## 5. Conclusion

Dynamic-enhanced MRI has high diagnostic sensitivity and specificity in axillary lymph node metastasis of breast cancer. The location, diameter, edge characteristics, early enhancement mode, and ADC value of breast cancer MRI are all related to axillary lymph node metastasis, and MRI is worthy of clinical application. There are still some shortcomings in this study, such as a small sample size and incomplete selection of research variables, which limit further research to a certain extent. In follow-up research, we should expand the sample size and conduct in-depth research and analysis in a large-sample, multi-center manner [13].

## Figures and Tables

**Figure 1:** Diagnostic ROC curve of axillary lymph node metastasis in breast cancer by MRI.

**Figure 2:** Multivariate logistic regression analysis of the characteristics of axillary lymph node metastasis in breast cancer.

**Table 1:** Results of pathological examination and MRI examination.

MRI	Pathological examination		Summation
	Shift	Not transferred	
Shift	92	10	102
Not transferred	8	90	98
Summation	100	100	200

**Table 2:** Diagnostic efficacy of MRI in breast cancer with axillary lymph node metastasis.

Check the plan	AUC	Standard error	Sensitivity	Specificity	*P*	95% CI
MRI	0.910	0.023	90.00	92.00	<0.001	0.864∼0.956

**Table 3:** Univariate analysis of the associations between breast cancer MRI findings and axillary lymph node metastasis (*n* = 100, %).

MRI expressions	Axillary lymph node metastasis group	Breast cancer alone group	*x * ^2^	*P*
Position			10.710	0.001
Exterior quadrant	67 (67.00)	44 (44.00)		
Internal quadrant	28 (28.00)	36 (36.00)		
Area centralis	5 (5.00)	20 (20.00)		
Type			1.987	0.159
Bossing	76 (76.00)	67 (67.00)		
Nonmass	24 (24.00)	33 (33.00)		

**Table 4:** Univariate analysis of the relationship between MRI features of breast lump-like lesions and axillary lymph node metastasis (*n* = 100, %).

MRI expressions	Axillary lymph node metastasis group	Breast cancer alone group	*x* ^2^	*P*
Form			0.981	0.322
Circular	45 (45.00)	52 (52.00)		
Oval	25 (25.00)	22 (22.00)		
Irregular shape	30 (30.00)	26 (26.00)		
Edge feature			13.569	<0.001
Smooth	34 (34.00)	60 (60.00)		
Irregular	66 (66.00)	40 (40.00)		
Internal reinforcement mode			0.533	0.465
Even	35 (35.00)	40 (40.00)		
Inhomogeneous	25 (25.00)	22 (22.00)		
Ring enhancement	40 (40.00)	38 (38.00)		
Early reinforcement mode			11.873	0.001
Slow strengthening	22 (22.00)	45 (45.00)		
Medium reinforcement	23 (23.00)	25 (25.00)		
Quick strengthening	55 (55.00)	30 (30.00)		
Maximum diameter (mm)	21.32 ± 6.78	16.74 ± 5.23	5.349	<0.001
ADC price (×10^−3^ mm^2^/s)	0.74 ± 0.29	0.91 ± 0.35	−3.740	<0.001

**Table 5:** Variable assignment table.

Indexes	Variable	Assignment
Position	*X*1	1 = exterior quadrant, 2 = internal quadrant, 3 = area centralis
Edge feature	*X*2	1 = irregular, 2 = smooth
Early reinforcement mode	*X*3	1 = slow strengthening, 2 = medium reinforcement, 3 = quick strengthening
ADC price	*X*4	—
Maximum diameter	*X*5	—
Axillary lymph node metastasis	*Y*	1 = yes, 2 = no

RETRACTED

**Table 6:** Multivariate logistic regression analysis of MRI imaging characteristics in breast cancer with axillary lymph node metastasis.

Parameters	*β*	Wald	*P*	OR (95% CI)
Position	0.877	12.267	<0.01	2.428 (1.477–3.989)

Edge feature	0.427	20.954	<0.01	0.641 (0.532–0.775)

Early reinforcement mode	0.963	17.214	<0.01	2.651 (1.669–4.195)

ADC price	-5.262	17.243	<0.001	0.009 (0.001∼0.062)

Maximum diameter	0.526	8.106	<0.01	1.706 (1.176–2.485)

## Data Availability

The simulation experiment data used to support the findings of this study are available from the corresponding author upon request.
